# Cerebrovascular Risk Factors in Possible or Probable Cerebral Amyloid Angiopathy, Modifier or Bystander?

**DOI:** 10.3389/fneur.2021.676931

**Published:** 2021-07-21

**Authors:** Andrea Wagner, Jonas Maderer, Sibylle Wilfling, Johanna Kaiser, Mustafa Kilic, Ralf A. Linker, Karl-Michael Schebesch, Felix Schlachetzki

**Affiliations:** ^1^Department of Neurology, University of Regensburg, Regensburg, Germany; ^2^Department of Neurosurgery, University Hospital Regensburg, Regensburg, Germany

**Keywords:** cerebral amyloid angiopathy, intracerebral hemorrhage, long term outcome, risk factors (cardiovascular) comorbidities, computer tomography, magnetic resonance imaging

## Abstract

**Goal:** Cerebral amyloid angiopathy (CAA) is a frequent cause of atypical intracerebral hemorrhage (ICH) in the elderly. Stroke risk factors such as arterial hypertension (AHT), atrial fibrillation (AFib), diabetes mellitus (DM), and renal dysfunction (RD) are increasingly apparent in these patients. In this retrospective study, we analyzed the presence of these stroke risk factors in different initial CAA presentations comprising cerebral microbleeds (CMB), acute ischemic stroke (AIS), cortical superficial hemosiderosis (cSS), or lobar ICH (LICH) and evaluated their influence on the initial clinical presentation of patients with CAA.

**Material and Methods:** We identified patients with at least possible CAA defined by the modified Boston criteria admitted to the Department of Neurology or Neurosurgery from 2002 to 2018.

**Findings:** In the overall cohort of 209 patients, we analyzed the correlation between the number of stroke risk factors and the initial clinical presentation of patients with CAA and could show the high multimorbidity of the collective. There are large differences between the subgroups with different initial clinical presentations, e.g., patients with CMB as initial CAA presentation have the highest number of cerebrovascular risk factors and recurrent AIS, whereas AFib is more frequent in the Neurosurgery Department.

**Conclusion:** There is a distinct overlap between the subgroups of CAA manifestations and stroke risk factors that need to be verified in larger patient collectives. Since these comorbidities are likely to influence the clinical course of CAA, they represent possible targets for secondary prevention until specific treatment for CAA becomes available.

## Introduction

Cerebral amyloid angiopathy (CAA) is a type 2 small vessel disease (SVD) and is responsible for up to 20% of non-traumatic intracerebral hemorrhages (ICH). It is surpassed only by type 1 SVD with its driving risk factors arterial hypertension (AHT) and diabetes mellitus (DM) (1–5). Currently, the only established genetic risk factors for CAA are apolipoprotein E ε2 and ε4 (1, 2, 4, 6–10). Since specific therapies for CAA do not exist, secondary prevention against recurrent CAA-related ICH is required as a strict antihypertensive management and the avoidance of additional cerebrovascular risk factors (1, 4, 8, 11, 12). Yet, the impact of established vascular risk factors on the development and course of CAA is still being investigated as the overlap with CAA increases with age. The current study aims to characterize the presence of vascular risk factors in different initial presentations of patients with at least possible CAA.

## Materials and Methods

The study was approved by the Ethical Review Board of the University of Regensburg (reference: 16-101-0050/16-050-101). The goal of the study was to address the question, whether single risk factors and the number of risk factors will influence the initial presentation of patients with at least possible CAA, which was subgrouped into LICH, AIS, CMB, and cSAH/cSS.

Discharge letters of patients treated in the Department of Neurology at the University of Regensburg or the Department of Neurosurgery at the University Hospital Regensburg between 2002 and 2018 were screened for the diagnosis of CAA according to the modified Boston criteria (13). According to the modified Boston criteria, patients in the LICH-group could also be included by cCT, if the modified Boston criteria were fulfilled. Patients of the other three groups were included on basis of cMRI (Figure 1).

**Figure 1:** Figure resuming data collection.

All available magnetic resonance imaging (MRI) data prior, during, or upon follow-up of the initial hospital stay were examined by trained study authors (AW and JK) who were blinded for the risk factors, and discussed where necessary with the neuroradiologic department for CMB using the MARS criteria (The Microbleed Anatomical Rating Scale criteria) and for cSAH/cSS, for correct classification of the patients into the subgroups (14, 15). cSS was further subgrouped in focal (less than four affected sulci) and disseminated cSS (more than four affected sulci) (16). In addition, we searched for recent ischemic lesions on diffusion-weighted imaging sequences, white matter hyperintensities (WMH) classified by the Fazekas score, residual lesions caused by previous AIS and ICH, and cerebral edema (17, 18). Classification of CAA in subtypes was performed according to the primary manifestation of CAA in the individual patient: patients with a (symptomatic) LICH were grouped into the LICH group, patients who got the diagnosis of CAA in an MRI for any other reason and showed multiple strictly lobar CMB (defined as >/= 5 CMB) were grouped into the CMB group, patients with symptomatic or asymptomatic cSS or a cSAH after exclusion of other reasons for cSAH were grouped into the cSS/cSAH group and patients who presented with an AIS proven by MRI who fulfilled diagnostic criteria for CAA were grouped into the AIS group.

To avoid misclassification of patients with only single CMBs as CAA, we defined a cutoff of >/=5 CMBs in accordance with Charidimou et al. (19) and Wilson et al. (20) as necessary for the diagnosis of CAA if other inclusion criteria like strictly lobar major ICH or cSS were lacking.

First, the following basic data were extracted from medical records for the index event: age and sex, symptoms at presentation, and AHT (first documented blood pressure at presentation, antihypertensive medication, or history of hypertension). A systolic blood pressure > 180 mmHg or diastolic blood pressure > 120 mmHg at first measurement (as assessed either by paramedics or in the emergency department) was defined as a hypertensive crisis. DM was defined as HbA1c > 6.5% (>58 mmol/mol) or preexisting antidiabetic medication and was subgrouped into insulin-dependent (IDM) and non-insulin-dependent (NIDM). Hypercholesterinemia was defined as LDL > 110 mg/dl or previous therapy with lipid-lowering drugs like statins or fibrates. The glomerular filtration rate (GFR), according to the Cockroft-Gault formula and therapy with diuretics were used to classify patients with renal insufficiency, with a GFR < 60 ml/min defined as renal failure. Cardiac comorbidities (defined as cardiac insufficiency, coronary heart disease, and cardiac arrhythmia) were recorded wherever possible. Furthermore, the diagnosis of AFib was evaluated from the records of patients, including electrocardiogram (ECG) monitoring results, if available. In patients with more than one contact to the Departments of Neurology or Neurosurgery, further, ICH/AIS were recorded.

To characterize the atherosclerotic load linked to the aforementioned vascular risk factors, we analyzed all available neurosonographic examinations and noted the diameter of the common carotid artery (CCA), intima-media thickness ratio, resistance index (RI) defined as RI = (S-D)/S (S = maximal systolic Doppler-frequency; D = maximal diastolic Doppler-frequency), and pulsatility index (PI) defined as PI = (S-D)/M (S = maximal systolic Doppler-frequency; D = maximal diastolic Doppler-frequency, M = mean velocity). In patients with unilateral stenosis of the internal carotid artery (ICA), classification according to the North Atlantic Carotid Artery Trial (NASCET) (21) was applied for assessment of the intima-media thickness ratio and RI of the contralateral ICA were used. Furthermore, the echogenicity of plaques in the common carotid artery (CCA) was graded from 1 to 4 as echolucent, predominantly echolucent, predominantly echogenic, or echogenic (22). Transthoracic echocardiography (TTE) was graded, wherever available in left ventricular hypertrophy (LVH), wall motion abnormalities, diastolic dysfunction, valvular sclerosis, valvular insufficiencies or stenoses, and reduced ejection fraction.

The percentage of risk factors for each patient subgroup was evaluated. Therefore, each of the seven possible risk factors [AHT, DM, atrial fibrillation (AFib), cardiac comorbidities, renal comorbidities, hypercholesterinemia, and hyperalbuminemia] in each patient was rated as present or absent. In the case of patients with several parameters missing, the percentage of present risk factors of patients with known risk factors was calculated, and this number was compared for the four subgroups.

Statistical analysis was done using Python's scipy.stats. For group comparisons, either two-tailed *t*-test, chi-square tests on contingency tables, or ANOVA were applied to the data as given in the text. *P* < 0.05 were considered significant. Data on subgroup analyses are available upon request.

## Results

Overall, we identified 209 patients with at least possible diagnosis of CAA according to the modified Boston criteria, 149 from the Department of Neurology, and 60 from the Department of Neurosurgery. Definite CAA was found in 15 patients, probable CAA with supporting pathology in 20 patients, probable CAA in 141 patients, and possible CAA in 33 patients. In the overall cohort, male and female patients were almost equally present (male 50.2%/105 patients, female 49.8%/104 patients), the average age was 72.32 years, with patients from the Department of Neurology slightly older than patients from the Department of Neurosurgery (73.05 vs. 70.50 years, two-sided *t*-test: *p* < 0.039), and women slightly older than men (73.3 vs. 71.4 years, non-significant, *p* > 0.094).

Due to the retrospective study design and the different diagnostical standard operating procedures in the Department of Neurology and Department of Neurosurgery, the information available on comorbidities and diagnostic procedures performed on the included patients were heterogeneous and partly incomplete. Thus, information about hypertension was available for 190 patients, HbA1c or diabetes for 206 patients, AFib for 201 patients, information on cardiovascular comorbidities in 203 patients, low-density lipoprotein (LDL) or medication for hypercholesterolemia for 188 patients, and intake of diuretics or GFR for diagnosis of chronic kidney disease in 190 cases.

All known cardiovascular comorbidities were registered on the admission of the patient as part of the anamnesis regardless of whether or not they were related to the acute symptomatic. These were in detail: coronary heart disease including those after coronary artery bypass graft or stent deployment, myocardial infarction, cardiac arrhythmia, heart failure, cardiac valve implantation, peripheral arterial occlusive disease including those after stent or bypass surgery, gastrointestinal ischemia, any stenosis or occlusion of brain supplying arteries including post carotid endarterectomy and stenting, ischemic or hemorrhagic stroke or transient ischemic attack, and renal insufficiency. Due to the retrospective study design only few patients had sufficient data on smoking, therefore we did not include that factor in our study.

Neurosonographic examination was available in 103 cases, TTE in 58 patients, and cMRI in 133 patients.

Regarding the primary manifestation of CAA, there were no significant differences based on sex (chi-square: *p* > 0.63). LICH was by far the most common primary manifestation (Figure 2) with a slight, non-significant higher percentage in women compared to men (*p* > 0.23 in chi-square).

**Figure 2:** The primary manifestation of cerebral amyloid angiopathy (CAA) in men vs. women such as lobar ICH (LICH), acute ischemic stroke (AIS), cerebral microbleeding (CMB), or cortical superficial hemosiderosis (cSS): Primary manifestation of CAA split by sex. The most common primary manifestation was ICB in both male and female patients. No significant differences could be found between the two sexes regarding primary manifestation (chi-square: *p* > 0.63). One male patient had both ICB and SAB/cSS and was counted to the ICB subgroup. The absolute numbers of patients are given above the bars. Percentages refer to the subgroup (all male patients, *n* = 105 and all female patients, *n* = 104).

Arterial hypertension as a comorbidity was extremely frequent in the patient with the CAA cohort. Only 15 of 190 patients did not fulfill the predefined criteria for the diagnosis of AHT at initial presentation resulting in a percentage of over 92%. No therapy with antihypertensive drugs was present in about 25% of patients with AHT at initial presentation (45/175).

With respect to the blood pressure at the initial presentation, no significant differences were found between the subgroups (ANOVA: *p* > 0.92). About one-third of the patients (58/164) with AHT showed hypertensive crisis (systolic blood pressure ≥180 mmHg) at initial presentation with a non-significant trend (chi-square: *p* > 0.83) toward more frequent hypertensive crises in the CMB (5/12 patients) and cSAH (5/11 patients) subgroups compared to LICH (38/113 patients) and AIS (10/28). In the overall cohort, 64/195 patients presented with hypertensive crisis.

Atrial fibrillation was frequent comorbidity with a lower incidence of 14.8% (21/142) in the neurological and a higher incidence of 28.8% (17/59) in the neurosurgical treated patients (chi-square contingency: *p* < 0.035). There were large differences between men (25.3% = 25/99 AFib) and women (12.7% = 13/102 AFib), with men being affected more frequently by AFib than women (*p* < 0.038 in chi-square). The incidence of AFib diverged largely between the subgroups: 21.4% of patients (31/145) with initial CAA manifestation with LICH, 25.0% of the cSS-subgroup (3/12), 10.3% of the AIS-subgroup (3/29), and 6.7% of the CMB-subgroup had AFib (1/15). The highest incidence of AFib of 30.3% was observed in men with ICH as a primary manifestation (20/66) (Figure 3).

**Figure 3:** Incidence of atrial fibrillation (AFib) in neurological vs. neurosurgical treated patients and men vs. women by index event.

### Risk Factor Hypercholesterinemia/Statin Therapy and CAA Subtypes

About one-third of patients (59/176) were treated with lipid-lowering therapy (i.e., statin or fibrate) at hospital admission, whereas only 39.6% (19/48) of the non-treated patients had a low-density-lipoprotein <110 mg/dl. Due to the retrospective study design and the small number of patients in the subgroups- only 59 patients of the whole collective took statins or another lipid-lowering medication, we decided not to perform subgroup analysis here.

### Risk Factor DM and Renal Insufficiency and CAA Subtypes: No Significant Influence of AHT on CAA Subtypes

38.4% (73/190) of patients suffered from renal insufficiency, defined as GFR (according to Cockroft-Gault) below 60 ml/min or intake of diuretics, and 20.5% (41/200) suffered from DM. 53.7% of patients with the diagnosis of DM (22/41) had IDM diabetes. Albuminuria was present in 33.0% (32/97 patients).

### Indications for Classical Cardiovascular Risk Factors by Technical Examinations- Neurosonographic Examination, TTE and Fazekas-Score in MRI

According to neurosonographic examination (104/209 patients), about one-fifth of patients (21/101) showed stenosis due to NASCET-criteria. Echogenicity was heterogeneous, with anechoic plaques (level 1–2) slightly more frequent (50/95) than echogenic plaques (level 3–4) (45/95) (Figure 4). In TTE, 61% (36/58) of patients had LVH or diastolic dysfunction. 39.4% of patients had a positive anamnesis of cardiological comorbidities (80/203). In 133 of 209 patients, MRI data were available. For 74/209 patients, clinical routine follow-up was available (Table 1). As a SVD marker, the Fazekas score was graded for periventricular white matter lesions (PWML-133 pat.) and deep white matter lesions (DWL-132 pat.) (Figure 5). For all subgroups, a Fazekas score of 0 was less common than a score of 1–3 without large differences between the subgroups.

**Figure 4:** Echogenity of plaques in neurosonographic examination.

**Table 1:** Patient characteristics.

**Department**	**Neuro-logic: 149**	**Neuro-surgical: 60**			
Sex	Female: 104	Male: 105			
Age (years)	MW: 72.32	STABWN: 8.06			
Primary manifestation	ICH: 151	AIS: 29	CMB: 16	cSAH/cSS: 13	
	Yes	No	Unknown		
Hypertension	175	15	19		
Hypertensive crisis	64	131	14		
Lipid-lowering therapy	59	117	33		
Hypercholesterinemia	80	29	100		
Diuretics	65	112	32		
Albuminuria	32	65	112		
Vascular comorbidity	80	123	6		
Atrial fibrillation	38	163	8		
MRI	133	76	0		
Follow-up (available only for patients of neurologic Department)	75	74	0		
Diabetes mellitus [no (n), (X), (u)]	iDM: 22	niDM: 14	No DM: 159	No known DM but HbA1c elevated justifying diagnosis of DM: 5	Un-known: 9
GFR (ml/min; <60, >60, u = unknown)	<60: 14	>60: 81	u: 114		

*Total number: 209; y, yes; n, no; u, unknown*.

**Figure 5:** Distribution of Fazekas scores among patients with CAA with MRI. Overall, a Fazekas score of 0 was less common than scores of 1–3 for both periventricular white matter lesions (PWML) and deep white matter lesions (DWL).

### High Percentage of Positive Classical Cardiovascular Risk Factors in CAA patients

On average, a patient showed 3.10/7 possible risk factors. The highest percentage of present risk factors was shown in the CMB group, with only slight differences between the different subgroups (average number of positive risk factors: ICH-group: 3.14/7; AIS-group: 2.75/7; CMB-group 3.36/7; cSAH-group: 3.25/7) (Figure 6).

**Figure 6:** Percentage of positive risk factors per subgroup.

## Discussion

There are large differences between the subgroups of CAA with a different initial presentation, which is well in accordance with previous studies (23–25). Primary ICH, in general, is more frequent in men (23, 26, 27). Patients with cSS are known to be an extremely vulnerable subgroup of patients with CAA with a high probability of recurrent ICH (28, 29). As almost 50% of those patients present with the hypertensive crisis in the emergency department, blood pressure management in this subgroup is a significant problem. The question arises whether the high number of hypertensive crises is a possible reason for symptomatic cSS or whether cSS is the reason for dysregulated high blood pressure.

The percentage of AHT at first presentation of CAA is far higher than the average frequency of about 46% in the overall adult population (30). Nevertheless, this high percentage might also be due to the older age within the CAA cohort compared to average adult age and, thus, cannot be compared directly with this population.

Patients show high potential for primary prevention by optimization of blood pressure management, e.g., by the general practitioners. Moreover, optimal blood pressure control is also a very important tool in secondary prophylaxis as good blood pressure management is known to be associated with less recurrent ICH, especially in patients with CAA (31, 32). Similar results are shown for the treatment of hypercholesterinemia, which was missing in about 60% of patients. This is higher than that to be expected compared with the general prevalence of elevated total cholesterol for a normal collective, which according to the WHO for the Region of Europe is 54% for both sexes^1^ In this research, the primary preventive potential is again high since patients not treated with lipid-lowering medication only reach a favorable LDL level of <110 mg/dl in 35% of cases. The incidence of DM (20%) at first sight is comparable with an age-matched normal collective^2^ However, the high discrepancy in the percentage of insulin-dependence in DM II between the literature (26%) (33) and our collective (50%) suggests a high number of unrecorded cases of NIDM, and therefore, a higher cumulative incidence of DM in our collective than in an age-matched normal collective. While the overall prevalence of chronic kidney disease in patients older than 20 years is 15% (30), in our older patient collective, we found a prevalence of any RD of 60%, which most likely is explained by age; and more prevalent diabetes and hypertension.

The high number of either pathologic findings in neurosonographic examination or TTE, the high Fazekas scores on MRI, and the high number of anamnestic cardiovascular comorbidities underpin the multimorbidity of the patient collective. The highest number of risk factors were found in the CMB-group, with 3.36/7 possible groups of risk factors positive vs. the other subgroups, with 3.10/7 possible groups of risk factors positive. This observation, together with our results of another study which showed that patients of that subgroup suffer the highest percentage of recurrent events in AIS (24), underlines that the CMB group, which is at first sight supposed to be mildly affected compared with patients presenting with a LICH, maybe the most vulnerable group of the collective. Indeed, patients with CMB may develop some type of protective mechanism like shifting of essential functions from the regions prone to bleed, which may also prevent further bleedings due to ongoing neuroplasticity, similar to patients with hemodynamically relevant stenosis of a cerebral vessel who suffer an AIS in the same region of the brain and are in part protected by ongoing collateral vessel formation (34). Due to the retrospective study design, in which patients with a second event were more likely to get a follow-up if CMB protects against a further ICH, the patients are more likely to get follow-up because of AIS. Yet, at the same time, the CMB group may harbor a high primary and secondary preventive potential.

The high number of concomitant cardiovascular risk factors fit the high Fazekas score as a marker for microvascular lesions. On the other hand, an interaction between WMH and CAA was already shown by the fact that patients with more WMH had a higher intensity of PiB (Pittsburgh compound B), showing amyloid β (35).

Excluding hypertension, the prevalence of chronic vascular disease (i.e., chronic heart disease, heart failure, and stroke) is 9.0% overall. A positive history of myocardial infarction was reported in 4.4% of patients, angina or chronic heart disease in 4.1%, and heart failure in 2.2% (30) of patients. In this research, the collective also shows a significantly higher prevalence as 39.4% of the patients had a positive history of cardiological comorbidities.

The large differences in the incidence of AFib between patients in the Neurological vs. Neurosurgical Department might be explained by the fact that patients with a large ICH or from a smaller clinic are more likely treated in the neurosurgery department, as the clinic as a tertiary referral center often gets patients transferred from smaller hospitals. Therefore, there might be a selection bias for worse cases toward the neurosurgery department. This observation is in line with a large study on ICH showing that patients with AFib-ICH were older and had more vascular risk factors, more antithrombotic pretreatment, a higher clinical severity, a higher hematoma volume, and higher in-hospital and 3-month mortality (36). The higher incidence of AFib in men is known from previous studies (37). We already proved AFib to be frequent in a cohort of patients with CAA treated in a neurosurgical ward (25.7%) with large differences between patients with probable CAA (4%), probable CAA with supporting pathology (33%), and possible CAA (38%) (25). In a neurological ward setting, the incidence of AFib (16%) is similar or only slightly higher than the cumulative incidence of AFib in other age-matched collectives (10–16%) (41, 42). AFib was shown to be reliable in predicting poor outcomes in primary ICH (38, 39). The higher cumulative incidence of AFib in neurosurgical treated patients with acute ICH may indicate a deeper relationship with CAA in the sympathetic brain-heart-axis, as already proposed by basic research (40).

## Strengths and Limitations

Due to retrospective study design, especially for patients with large LICH and primary palliative care concepts, datasets in some cases are incomplete. For example, in 15 patients, data with the information whether or not the patient is suffering from AHT is lacking. Especially in patients with a primary poor prognosis and palliative procedure, often, only basic data are available. The information on IDM might also be biased, as it is more likely to be recorded in patients with less information than those with information on oral medication.

A strength of this study is that we included and compared patients of neurological as well as neurosurgical ward and therefore have less selection bias, supposing that patients with larger bleedings are more often treated in the neurosurgical ward and vice versa.

## Summary

Cerebral amyloid angiopathy as an important cause of LICH is attracting increasing attention. Its frequency is increasing with an aging population. Overlap of CAA and classical cardiovascular comorbidities is high. While the prevalence of AFib with 16% is only slightly higher than that in an age-matched normal collective, AHT is extremely frequent with a prevalence >90%. There are large differences in the risk factors between the subgroups with different initial clinical presentations and clinical follow-ups also. The high number of concomitant cerebrovascular risk factors in patients with CAA, and the fact that there are large differences for these between the subgroups with a different initial presentation of CAA, makes it highly probable that the risk factors are not only bystanders but also modifiers. These data should be verified in a larger patient collective.

## Data Availability Statement

The raw data supporting the conclusions of this manuscript will be made available by the authors, without undue reservation, to any qualified researcher.

## Ethics Statement

The studies involving human participants were reviewed and approved by Ethical Review Board of the University of Regensburg. Written informed consent for participation was not required for this study in accordance with the national legislation and the institutional requirements.

## Author Contributions

AW, JM, SW, K-MS, and FS contributed to the conception and design of the study and analysis and interpretation of the data. AW and FS wrote the first draft of the manuscript. JM and SW contributed to analysis and interpretation of the data and wrote parts of the manuscript. JM, SW, JK, MK, K-MS, and RL wrote sections of the manuscript. All authors contributed to manuscript revision, read, and approved the submitted version.

## Conflict of Interest

The authors declare that the research was conducted in the absence of any commercial or financial relationships that could be construed as a potential conflict of interest.

## Footnotes

^1^https://www.who.int/gho/ncd/risk_factors/cholesterol_text/en/

^2^https://www.escardio.org/Education/Diabetes-and-CVD/Recommended-Reading/global-statistics-on-diabetes

## Abbreviations

ACC: common carotid artery
AFib: atrial fibrillation
AHT: arterial hypertension
AIS: acute ischemic stroke
CAA: cerebral amyloid angiopathy
CCA: common carotid artery
CMB: cerebral microbleeding(s)
cSAH: cortical subarachnoid hemorrhage
cSS: cortical superficial hemosiderosis
DM: diabetes mellitus
DWL: deep white matter lesions
ECG: electrocardiogram
GFR: glomerular filtration rate
ICA: internal carotid artery
ICH: intracerebral hemorrhage
IDM: insulin-dependent DM
LDL: low-density lipoprotein
LICH: lobar ICH
LVH: left ventricular hypertrophy
MARS criteria: The Microbleed Anatomical Rating Scale criteria
MRI: magnetic resonance imaging
NASCET: North Atlantic Carotid Artery Trial
NIDM: non-insulin-dependent DM
PI: pulsatility index
PiB: Pittsburgh compound B
PWML: periventricular white matter lesions
RD: renal dysfunction
RI: resistance index
SVD: small vessel disease
TTE: transthoracic echocardiography
WMH: white matter hyperintensities.
